# Clinical Relevance and Prognostic Value of the Neuronal Protein Neuroligin 2 in Breast Cancer

**DOI:** 10.3389/fonc.2021.630257

**Published:** 2021-11-03

**Authors:** Gang Zhang, Yi Sun, Zheng-sheng Wu, Xing Huang

**Affiliations:** ^1^ Zhejiang Provincial Key Laboratory of Pancreatic Disease, The First Affiliated Hospital, School of Medicine, Zhejiang University, Hangzhou, China; ^2^ Department of Pathology, Anhui Medical University, Hefei, China; ^3^ The Key Laboratory of Developmental Genes and Human Disease, Institute of Life Sciences, Southeast University, Nanjing, China

**Keywords:** neuroligin 2, cancer biomarker, breast cancer, clinical relevance, prognostic factor, cancer immunity, mitochondria

## Abstract

Neuroligin 2 (NLGN2) is a well-recognized transmembrane scaffolding protein that functions in synapse development and neuronal signal transduction. It has recently been implicated in multiple diseases of peripheral ectodermal origin. However, the potential roles of NLGN2 in tumors remain ill-defined. The aim of this study was to determine the clinical relevance and prognostic value of NLGN2 in breast cancer. To this end, breast cancer datasets were extracted from TCGA and other public databases, and subjected to Kaplan-Meier potter for survival analysis, GEPIA2 for assessing the immunological relevance of NLGN2 and THPA for identifying its subcellular localization. The *in-silico* results were further validated by immunohistochemistry analysis of *in-house* tumor tissue specimens. NLGN2 was identified as a prognostic factor in breast cancer subtypes, and its high expression correlated to a favorable survival outcome. Moreover, NLGN2 overexpression in breast cancer was significantly associated with large tumor size, lymph node metastasis, late TNM stage, and high histological grade. Interestingly, there was a significant correlation between the expression level of NLGN2 and the immunomodulatory molecules, along with increased interstitial infiltration of lymphocytes. Furthermore, NLGN2 was predominantly localized in the mitochondria of breast cancer cells. In conclusion, NLGN2 has a prognostic role and immunoregulatory potential in breast cancer, and its functions likely have a mitochondrial basis. It is a promising therapeutic target in breast cancer and should be explored further.

## Introduction

The incidence of breast cancer has increased steadily from 2005 to 2016 due to a combination of lifestyle-related factors and genetic predisposition (1, 2). It currently accounts for 30% of all newly diagnosed cancers, and is the leading cause of cancer-related mortality among females (3). Notwithstanding, the death rate of breast cancer continues to decline, and dropped to 40% in the period between 1989 and 2017, and averted an estimated 375900 breast cancer-related deaths in the United States (4). This trend is largely attributed to the early diagnosis and novel therapeutic strategies that consider the inherent molecular heterogeneity between individual patients (5). In fact, ~70-80% breast cancer patients present with early-stage disease that is either confined to the breast or spread to the axillary lymph nodes, and is considered curable. The prognoses of the remaining metastatic patients have also improved considerably due to locoregional and systemic therapies targeted against the specific subtypes that are classified on the basis of both histological and molecular characteristics, including triple-negative, HER2-enriched non-luminal, luminal B-like HER2+, luminal B-like HER2-, and luminal A-like subjects (5, 6). Nevertheless, the existing treatment strategies cannot completely cure the metastatic subtype even after improving patient survival. Studies increasingly show that the immune system greatly influences therapeutic efficacy and patient prognoses (5). The immune microenvironment consisting of activated CD8+ and CD4+ T cells exert an anti-cancer role during tumor initiation but turn pro-tumorigenic during invasive growth. Therefore, in addition to the established prognostic markers (e.g., p-STAT3, HER2 and LDH) have of breast cancer (7–9), immunologically favorable biomarkers are also needed to guide the choice and administration of therapeutic strategy for breast cancer patients.

Neuroligin 2 (NLGN2) is an important post-synaptic neural cell adhesion protein and the only member of the neuroligin family that functions exclusively at GABAergic inhibitory synapses (10). The neurological functions of NLGN2 are well documented, and mainly depend on its interactions with the members of the neurexin (NRXN) family (11–15). The trans-synaptic interactions of NLGN2 with NRXNs, as well as the postsynaptic interactions with Cb and gephyrin, recruit GABA_A_Rs and gephyrin to the synapses, which regulates the formation and strength of inhibitory synapse and balances the inhibitory and excitatory neuronal networks (10, 12). Mutations and genetic variations in NLGN2 are related to several neurocognitive diseases, such as motor incoordination, social impairment, aggression, schizophrenia, anxiety, depression and intellectual disability (11, 16–18). For instance, the local removal of NLGN2 from adult medial prefrontal cortex neurons decreased inhibitory synaptic transmission, resulting in considerable behavioral impairment. Moreover, functional knockdown of NLGN2 in dopamine D1-positive cells facilitated subordination and stress susceptibility, while that in dopamine D2-positive cells regulated active defensive behavior. Interestingly, there is emerging evidence of non-neurological functions of NLGN2 in the peripheral tissues. For instance, Zhang et al. reported that the NLGN2 expressed on pancreatic beta-cells promotes normal insulin secretion through transcellular interactions (19). Pergolizzi et al. found that NLGN2 expressed in vascular endothelial cells regulates angiogenesis by inducing release of vascular factors (20). In addition, Yang et al. showed that down-regulation of NLGN2 in the ganglion colon segment is associated with excessive intestinal contraction and increased risk of Hirschsprung disease (21). However, the potential involvement of NLGN2 in peripheral tumors remains poorly identified so far.

In this study, we analyzed the potential role of NLGN2 in breast cancer, which is under partial neuroendocrine neoplastic growth. We assessed the expression levels and prognostic values of NLGN2 in the open-access genome and proteome datasets of breast cancer, and validated the *in-silico* bioinformatics results with *in-house* patient tissue samples. We also investigated the role of NLGN2 in the overall survival of patients with different breast cancer subtypes, its correlation with local immunomodulatory molecules and cells, as well as its intracellular localization.

## Materials and Methods

### Patient Tissue Sample Collection

One hundred paraffin-embedded breast tumor specimens were collected from patients that underwent surgery at the First Affiliated Hospital of Anhui Medical University (Hefei, Anhui, China) between 2017 and 2021. The acquisition of patient tissue samples and all procedures used in this study were approved by the Ethics Committee of Anhui Medical University. Informed consent was obtained from each patient, and the specimen usage was in line with the Declaration of Helsinki.

### Kaplan-Meier Survival Analysis

The prognostic value of NLGN2 in breast cancer was assessed with the Kaplan-Meier Plotter (KM Plotter, http://kmplot.com/analysis) (22), an online database with gene expression profiles and overall survival (OS) data of cancer patients. The respective patient cohorts, including 1764 cases of breast cancer available on KM Plotter, were divided into the NLGN2^high^ and NLGN2^low^ groups based on the median mRNA expression levels, and their survival rates and duration were analyzed using the Kaplan-Meier survival plots. Hazard ratio (HR), 95% confidence interval (95% CI) and log-rank *p* value were calculated, and *p* < 0.05 was considered statistically significant.

### Gene Expression Profiling Interactive Analysis

The correlations between NLGN2 expression and multiple immune signatures were assessed by Gene Expression Profiling Interactive Analysis (GEPIA, http://gepia2.cancer-pku.cn, version 2) (23). The raw RNA-Seq data downloaded from TCGA and GTEx databases were processed with the UCSC Xena project following a standard analysis pipeline to avoid data imbalance and ineffective differential analyses. The pair-wise correlations were calculated by Spearman analysis, and *p* < 0.05 was considered statistically significant.

### Immunohistochemistry Analysis

The *in-situ* expressions of NLGN2, CD3 and CD8 proteins in paraffin-embedded breast tumor tissue sections were examined by immunohistochemistry as previously described (24) with rabbit anti-NLGN2 (1:200, bs-11098R, Bioss), anti-CD3 (1:1000, 60181-1-Ig, Proteintech) and anti-CD8 (1:1000, 66868-1-Ig, Proteintech) polyclonal antibodies. Five random fields were viewed per slide under high power. The NLGN2 staining intensity in the tumor cells (graded 0–3) and the percentage of stained cells (0 - no tumor cells positive; 1 - 10%–25% positive cells, 2 - 25%–50%, and 3 > 50%) were recorded, and multiplied to obtain the staining index ranging from 0 to 9 (25). Samples with staining indices 0-3 and >3 were designated as NLGN2^low^ and NLGN2^high^, respectively. The number of infiltrating CD3 and CD8 positive cells in the tumor stroma were scored (1 - 0 ~ 25, 2 - 26 ~ 50, 3 - 51 ~ 75, and 4 > 75) at 400× final magnification (26), and the samples were classified as low expressing and high expressing based on positive cell count of 1 and 2 ~ 4 respectively.

### Subcellular Location Analysis by THPA

The NLGN2 immunofluorescence images of multiple cell lines were acquired from The Human Protein Atlas (THPA, http://www.proteinatlas.org) (27), after authorization by the HPA team for the use for specific and scientific publication.

### Statistical Analysis

SPSS22.0 was used for data analysis. Chi-square test was used to compare variables, and the correlation between factors was assessed by the Spearman method. *P* < 0.05 was considered statistically significant.

### Availability of Data and Materials

The results shown in this study are based on TCGA Research Network (https://www.cancer.gov/tcga), THPA (v18.1.proteinatlas.org), and IHC staining. All datasets analyzed during the current study are available in TCGA (http://cancergenome.nih.gov) and THPA (http://www.proteinatlas.org). All other data generated during the current study are included in this published article. Further information is available from the corresponding authors upon reasonable request.

## Results

### NLGN2 Overexpression Is Favorable for the Survival of Breast Cancer Patients

To determine the prognostic relevance of NLGN2 in breast cancer, patients from multiple breast cancer datasets (totally 1764 subjects) were classified into the NLGN2^high^ and NLGN2^low^ groups, and their survival was analyzed using KM Plotter (28). As shown in **Figure 1A**, the NLGN2^high^ patients had significantly longer overall survival compared to the NLGN2^low^ group (HR, 0.59; 95%CI, 0.5 to 0.69; *p* < 0.05), including those post-treated (HR, 0.51; 95%CI, 0.41 to 0.64; *p* < 0.05) **(** **Figure 1B** **)**. The favorable prognostic function of NLGN2 was also confirmed for the basal (HR, 0.72; 95%CI, 0.52 to 1; *p* < 0.05) **(** **Figure 1C** **)**, luminal A (HR, 0.65; 95%CI, 0.5 to 0.83; *p* < 0.05) **(** **Figure 1D** **)**, and luminal B (HR, 0.54; 95%CI, 0.39 to 0.73; *p* < 0.05) **(** **Figure 1E** **)** subtypes. In contrast, higher expression of NLGN2 was not conductive to the survival of the HER2+ breast cancer patients (HR, 0.59; 95%CI, 0.5 to 0.69; *p* > 0.05) **(** **Figure 1F** **)**. Taken together, unlike the currently established breast cancer biomarkers, elevated NLGN2 indicates favorable prognosis for breast cancer patients with the basal, luminal A, and luminal B phenotypes.

**Figure 1:** NLGN2 is a prognostic factor of breast cancer. **(A)** Prognostic analysis of NLGN2 in breast cancer. **(B)** Prognostic analysis of NLGN2 in post-treated breast cancer. **(C)** Prognostic analysis of NLGN2 in basal breast cancer. **(D)** Prognostic analysis of NLGN2 in luminal A breast cancer. **(E)** Prognostic analysis of NLGN2 in luminal B breast cancer. **(F)** Prognostic analysis of NLGN2 in HER2+ breast cancer. The HR and log rank *p* values are indicated in each panel, and *p* < 0.05 is statistically significant.

### The Prognostic Value of NLGN2 for Specific Molecular Subtypes of Breast Cancer

To further determine the clinical pertinence of NLGN2 in breast cancer, we assessed its prognostic performance in different intrinsic subtypes with or without the estrogen receptor (ER), progesterone receptor (PR) and Erb-B2 receptor tyrosine kinase 2 (HER2) expression. NLGN2 overexpression was not associated with prognosis in the ER negative (-) patients (HR, 0.97; 95%CI, 0.7 to 1.36; *p* > 0.05) **(** **Figure 2A** **)** and PR- patients (HR, 1.07; 95%CI, 0.75 to 1.53; *p* > 0.05) **(** **Figure 2B** **)**. In contrast, elevated NLGN2 expression was related to prolonged survival in HER2- patients (HR, 0.7; 95%CI, 0.52 to 0.95; *p* < 0.05) **(** **Figure 2C** **)**, which was not observed in the ER-/PR-/HER2- patients (HR, 1.18; 95%CI, 0.68 to 2.04; *p* > 0.05) **(** **Figure 2D** **)**. In addition, there was no significant correlation between NLGN2 and OS in patients with wild type tumor protein p53 (TP53) (HR, 1.46; 95%CI, 0.63 to 3.42; *p* > 0.05) **(** **Figure 2E** **)** or mutated TP53 (HR, 0.87; 95%CI, 0.48 to 1.58; *p* > 0.05) **(** **Figure 2F** **)**. Thus, the upregulation of NLGN2 is associated with better prognosis in HER2- breast cancer as opposed to other molecular subtypes.

**Figure 2:** NLGN2 is favorable for HER2- breast cancer patients. **(A)** Prognostic analysis of NLGN2 in ER- breast cancer. **(B)** Prognostic analysis of NLGN2 in PR- breast cancer. **(C)** Prognostic analysis of NLGN2 in HER2- breast cancer. **(D)** Prognostic analysis of NLGN2 in ER-/PR-/HER2- breast cancer. **(E)** Prognostic analysis of NLGN2 in TP53 wild type breast cancer. **(F)** Prognostic analysis of NLGN2 in TP53 mutated breast cancer. The HR and log rank *p* values are indicated in each panel, and *p* < 0.05 is statistically significant.

### NLGN2 Is a Favorable Biomarker in Breast Cancer Patients Without Tumor Lymph Node Metastasis

Given the relevance of tumor metastasis and pathological grading in the survival of breast cancer patients, we next analyzed the relationship between NLGN2 expression and the status of tumor lymph node metastasis or tumor grades. NLGN2 was identified as a favorable prognostic factor in the tumor lymph node non-metastatic (-) patients (HR, 0.65; 95%CI, 0.44 to 0.97; *p* < 0.05) **(** **Figure 3A** **)**, but not in the tumor lymph node metastatic (+) patients (HR, 0.92; 95%CI, 0.72 to 1.19; *p* > 0.05) **(** **Figure 3B** **)**. Surprisingly, the expression of NLGN2 was not correlated with the survival of patients diagnosed as Grade 1 (HR, 0.73; 95%CI, 0.25 to 2.1; *p* > 0.05) **(** **Figure 3C** **)**, Grade 2 (HR, 1.18; 95%CI, 0.71 to 1.97; *p* > 0.05) **(** **Figure 3D** **)** and Grade 3 (HR, 0.81; 95%CI, 0.6 to 1.11; *p* > 0.05) **(** **Figure 3E** **)**. Taken together, NLGN2 expression correlates to the metastasis of breast cancer as opposed to pathological grading.

**Figure 3:** NLGN2 is favorable in lymph node non-metastatic breast cancer patients. **(A)** Prognostic analysis of NLGN2 in lymph node- breast cancer. **(B)** Prognostic analysis of NLGN2 in lymph node+ breast cancer. **(C)** Prognostic analysis of NLGN2 in Grade 1 breast cancer. **(D)** Prognostic analysis of NLGN2 in Grade 2 breast cancer. **(E)** Prognostic analysis of NLGN2 in Grade 3 breast cancer. The HR and log rank *p* values are indicated in each panel, and *p* < 0.05 is statistically significant.

### NLGN2 Positively Correlates With the Immunomodulatory Signature in Breast Cancer

Since immune regulation is a key factor in cancer progression, we also analyzed the potential influence of NLGN2 on breast cancer immunity to better understand its prognostic role. Intriguingly, NLGN2 expression was closely related to levels of critical immune effector molecules, including IFNG **(** **Figure 4A** **)** and GZMB **(** **Figure 4B** **)**. At the cellular landscape, NLGN2 correlated significantly with signatures of crucial subpopulations of tumor-infiltrating lymphocytes (29), including but not limited to cytotoxic T cells (CD3/CD8) **(** **Figure 4C** **)**, helper T cells (CD3/CD4) **(** **Figure 4D** **)**, B cells (CD19/CD20) **(** **Figure 4E** **)**, macrophages (CD14/CD11b/HLA-DR) **(** **Figure 4F** **)**, NK cells (CD16/CD56/NKG2D) **(** **Figure 4G** **)**, and dendritic cells (CD135/Flt3/CD117/CD26/CD103) **(** **Figure 4H** **)**. Taken together, these findings indicated that NLGN2 might have an immune system-dependent role in breast cancer, and the prognostic significance of NLGN2 is likely due to its correlation with a favorable immune signature.

**Figure 4:** NLGN2 correlates with immune signatures in breast tumor. **(A)** Correlation analysis of NLGN2 and IFNG in breast cancer (BRCA). **(B)** Correlation analysis of NLGN2 and GZMB in BRCA. **(C)** Correlation analysis of NLGN2 and Cytotoxic T cell signatures in BRCA. **(D)** Correlation analysis of NLGN2 and Helper T cell signatures in BRCA. **(E)** Correlation analysis of NLGN2 and B cell signatures in BRCA. **(F)** Correlation analysis of NLGN2 and Macrophage cell signatures in BRCA. **(G)** Correlation analysis of NLGN2 and NK cell signatures in BRCA. **(H)** Correlation analysis of NLGN2 and Dendritic cell signatures in BRCA. The *p* values and R coefficient are indicated in each panel, and *p* < 0.05 is statistically significant.

### Expression of NLGN2 Is Associated With Clinicopathological Features and Tumor Infiltrating CD3+ and CD8+ T Lymphocytes in Breast Cancer

To validate the *in-silico* prognostic data of NLGN2 in breast cancer, we next analyzed its *in-situ* expression levels in patient tissue samples by IHC staining. NLGN2 was highly expressed in 75% (75/100) of the tumor samples, and its expression level was significantly associated with tumor size, lymph node metastasis, TNM stage and histological grade (all *p* < 0.05), but not with patient age or the expression levels of ER, PR and HER2 (all *p* > 0.05) **(** **Figure 5** and **Table 1** **)**. To determine the correlation between NLGN2 and lymphocytes infiltration, the tumor tissues with differential NLGN2 expression were immuno-stained with anti-CD3 and anti-CD8 polyclonal antibodies. As shown in **Figure 5** and **Table 2**, 82.7% (62/75) and 74.7% (56/75) of the NLGN2^high^ samples had an abundance of CD3+ and CD8+ cells infiltration, while 44% (11/25) and 72% (18/25) of the NLGN2^low^ samples showed significantly decreased CD3+ and CD8+ T cell infiltration, respectively. Thus, NLGN2 expression was significantly correlated with the interstitial infiltration of both CD3+ and CD8+ T lymphocytes (both *p* < 0.01). These findings further underscore the close association between NLGN2 expression in breast cancer and the clinicopathological features as well as lymphocytes infiltration.

**Figure 5:** Association of the expression levels of NLGN2, CD3 and CD8 in breast cancer. Representative images of immunohistochemical staining showing *in situ* expression of NLGN2, CD3 and CD8 in breast cancer tissue specimens. Left panels, low expression of NLGN2 in breast tumor tissue, and CD3+ and CD8+ T cells in the same tissue. Right panels, high expression of NLGN2 in breast tumor tissue, and CD3+ and CD8+ T cells in the same tissue. The arrows point to CD3+ or CD8+ lymphocytes. All photos are at 400× original magnification.

**Table 1:** The relationship between NLGN2 expression and the clinicopathological features of breast cancer patients.

Parameter	n	NLGN2		*P* value
		Low expression	High expression	
**Age (years)**				0.63
**< 50**	36	10 (27.8%)	26 (72.2%)	
**≥ 50**	64	15 (23.4%)	49 (76.6%)	
**Tumor size (cm)**				0.01
**< 5**	85	23 (27.1%)	62 (72.9%)	
** ≥ 5**	15	2 (13.3%)	13 (86.7%)	
**Lymph node metastasis**				0.03
**+**	38	5 (13.2%)	33 (86.8%)	
**-**	62	20 (32.3%)	42 (67.7%)	
**Grade**				0.02
** I and II**	64	21 (32.8%)	43 (67.2%)	
** III**	36	4 (11.1%)	32 (88.9%)	
**Stage**				< 0.01
** I and II**	77	11 (14.3%)	66 (85.7%)	
** III**	23	14 (60.9%)	9 (39.1%)	
**ER**				0.08
** +**	70	14 (20.0%)	56 (80.0%)	
**-**	30	11 (36.7%)	19 (63.3%)	
**PR**				0.19
** +**	63	13 (20.6%)	50 (79.4%)	
**-**	37	12 (32.4%)	25 (67.6%)	
**Her-2**				0.13
** 0 ~ 1 +**	43	14 (32.6%)	29 (67.4%)	
** 2 + ~ 3 +**	57	11 (19.3%)	46 (80.7%)	

ER, PR, and HER2 data were obtained from patients’ pathology records.

**Table 2:** The relationship between NLGN2 expression and CD3+ and CD8+ tumor infiltrating lymphocytes.

	n	Tumor infiltrating CD3+ lymphocyte		*P* value	Tumor infiltrating CD8+ lymphocyte		*P* value
		Low level	High level		Low level	High level	
**NLGN2**				< 0.01			< 0.01
**Low expression**	25	11 (44.0%)	14 (56.0%)		18 (72.0%)	7 (28.0%)	
**High expression**	75	13 (17.3%)	62 (82.7%)		19 (25.3%)	56 (74.7%)	

### NLGN2 Is Located in the Mitochondria of Peripheral Breast Cancer Cells

As shown in **Figure 5**, the CD3+ and CD8+ lymphocytes were mainly distributed in the interstitial tissue, whereas NLGN2 was primarily localized in the cytoplasm rather than the plasma membrane of normal and malignant breast epithelial cells. Since the spatial distribution of a protein is a determinant of its function and mechanism, we further assessed the distribution of NLGN2 in breast cancer cells using the THPA database based on integrated multiple analyses (27). Interestingly, NLGN2 expression was predominantly localized in the mitochondria of the MCF7 breast cancer cell line **(** **Figure 6A** **)**. Moreover, the unusual positioning of NLGN2 in mitochondria was also observed in several other tumor and normal cell lines, including U2OS **(** **Figure 6B** **)**, U251MG **(** **Figure 6C** **)** and NIH3T3 **(** **Figure 6D** **)**. Mitochondrion is a major determinant of cancer cell growth and patient survival due to its pivotal roles in metabolite transport, energy production, apoptosis induction, and the immune stimulation (30). We therefore hypothesize that the mitochondrial localization of NLGN2 is instrumental to its prognostic role in breast cancer, and should be explored further, especially from the perspectives of immunoregulation and immunotherapy.

**Figure 6:** NLGN2 is localized in the mitochondria of multiple cancer and normal cells. **(A–D)** Representative immunofluorescence images showing NLGN2 localization in **(A)** MCF7 breast adenocarcinoma cells, **(B)** U2OS osteosarcoma cells, **(C)** U251MG glioblastoma cells, and **(D)** NIH3T3 mouse embryonic fibroblast cells. Green: NLGN2; Blue: Nucleus.

## Discussion

Studies increasingly show neurological involvement in cancer onset and progression, and the nascent field of cancer neurobiology is a promising avenue for the development of innovative cancer therapeutic strategies (31). Peripheral neurotransmitter signals have been reported to regulate the development of pancreatic, colon, gastric, breast, prostate, oral, head and neck, glioma, ovary as well as skin tumors in preclinical models through direct or indirect interactions with the tumor or its microenvironment (31, 32). For example, the microenvironmental synapse protein NLGN3 stimulates glioma growth by activating multiple oncogenic pathways (e.g., focal adhesion kinase activated upstream of PI3K-mTOR) and inducing transcriptional changes (e.g., upregulation of synapse-related genes in glioma cells) (33, 34). In addition, the L1 cell adhesion molecule (L1CAM), an axonal glycoprotein involved in neuronal migration and differentiation, was recently identified as an oncogene that is overexpressed in colon and ovarian cancers, and associated with increased invasion and poor prognosis (35–37). Through *in-silico* assessment and further validation, we found here that the neuronal protein NLGN2 has significant clinical relevance and prognostic value in breast cancer. NLGN2 is upregulated in breast tumor tissues and correlates with higher survival rates. More importantly, to the best of our knowledge, this is the first study to demonstrate the mitochondrial location of NLGN2 and its association with immune signatures.

Mitochondria are the bioenergetic and metabolic centers of eukaryotic cells (38, 39), and regulate their proliferation, differentiation and death (40, 41). In addition, metabolic alterations in the mitochondria affect catabolic processes like apoptosis, autophagy and necrosis in cancer cells (42). Recent studies show that the mitochondria influence both innate and adaptive immune responses during tumor onset or progression by regulating T cell activation, memory CD8+ cell formation, CD4+ T cell differentiation, B cell function, macrophage polarization, dendritic cells and inflammasome activation (40, 41, 43). However, metabolic reprograming of tumor cells leads to hypoxia and nutrient deficiency in the tumors, thereby triggering mitochondrial dysfunction in the immune cells and impairing their functions (40). Restoring glycolysis in the context of glucose deprivation boosts anticancer response of the tumor infiltrating lymphocytes. Prolyl hydroxy lase2­deficient T cells with increased glycolytic activity due to HIF1α stabilization showed stronger tumoricidal effects compared to their wild­type counterparts. In addition, the deficiency of peroxisome proliferator-activated receptor γ coactivator-1 (PGC1α) in multiple cancers (e.g., colon and breast cancer) impairs mitochondrial biogenesis in the infiltrating T cells, leading to mitochondrial dysfunction and reduced T cell-mediated cytotoxicity (40, 44). The anti-tumor effects of these T cells can be restored by rescuing mitochondria *via* ectopic PGC1α expression. In another study, adoptively transferred melanoma-specific CD8+ T cells induced a stronger anti-cancer response following selective removal of cells with low mitochondrial membrane potential. These findings suggest that mitochondrial dysfunction of immune cells can be reversed by restoring cancer cell metabolism, resulting in improved function and infiltration. Accordingly, it is rational to surmise that the mitochondrial location of NLGN2 is critical for its prognostic role in breast cancer, and the close association between NLGN2, mitochondria and immune signatures in breast cancer indicates that NLGN2 may play an immunoregulatory role by reversing mitochondrial dysfunction. Of note, we concluded the immunological relevance of NLGN2 in breast cancer solely through immunohistochemical staining of CD3+ and CD8+ T cells in the tumor tissues. Therefore, the comprehensive relationship between NLGN2 and immunological changes in the tumor microenvironment, as well as the mechanisms underlying mitochondrial involvement, remain to be elucidated by further gain or loss-of-function assays.

## Conclusions

NLGN2 expression level in breast tumors is associated with molecular subtypes, metastatic statues, immunomodulatory signatures and lymphocyte infiltration. The prognostic role of NLGN2 may be attributed to its mitochondrial location, and the mechanism warrants further investigation to consider NLGN2-targeted therapeutic strategy against breast cancer.

## Data Availability Statement

The original contributions presented in the study are included in the article/supplementary material. Further inquiries can be directed to the corresponding authors.

## Ethics Statement

The studies involving human participants were reviewed and approved by Ethics Committee of Anhui Medical University. The patients/participants provided their written informed consent to participate in this study.

## Author Contributions

XH conceived this study. XH, GZ, and YS collected the data. XH and Z-sW analyzed and interpreted the data. XH and GZ wrote and revised the manuscript. YS and Z-sW discussed the manuscript and provided inputs. GZ and YS contributed equally to the study. XH and Z-sW supervised the study and share the senior authorship. All authors contributed to the article and approved the submitted version.

## Funding

This study was funded by grants from the National Natural Science Foundation of China (31970696 and 81502975 to XH; 81972472 to Z-sW), China Postdoctoral Science Foundation (2016T90413 and 2015M581693 to XH), and Natural Science Foundation of Anhui (2008085MH276 to Z-sW).

## Conflict of Interest

The authors declare that the research was conducted in the absence of any commercial or financial relationships that could be construed as a potential conflict of interest.

## Publisher’s Note

All claims expressed in this article are solely those of the authors and do not necessarily represent those of their affiliated organizations, or those of the publisher, the editors and the reviewers. Any product that may be evaluated in this article, or claim that may be made by its manufacturer, is not guaranteed or endorsed by the publisher.

## Abbreviations

NLGN2, neuroligin 2; NRXN, neurexin; KM Plotter, Kaplan-Meier Plotter; OS, overall survival; HR, hazard ratio; GEPIA, Gene Expression Profiling Interactive Analysis; THPA, The Human Protein Atlas; ER, estrogen receptor; PR, progesterone receptor; HER2, Erb-B2 receptor tyrosine kinase 2; TP53, tumor protein p53; L1CAM, L1 cell adhesion molecule; peroxisome proliferator-activated receptor γ coactivator-1, PGC1α.
